# Multiparametric Magnetic Resonance Imaging Information Fusion Using Graph Convolutional Network for Glioma Grading

**DOI:** 10.1155/2022/7315665

**Published:** 2022-05-10

**Authors:** Peiying Guo, Longfei Li, Cheng Li, Weijian Huang, Guohua Zhao, Shanshan Wang, Meiyun Wang, Yusong Lin

**Affiliations:** ^1^School of Computer and Artificial Intelligence, Zhengzhou University, Zhengzhou 450001, China; ^2^Collaborative Innovation Center for Internet Healthcare, Zhengzhou University, Zhengzhou 450052, China; ^3^Paul C. Lauterbur Research Center for Biomedical Imaging, Shenzhen Institute of Advanced Technology, Chinese Academy of Sciences, Shenzhen 518000, China; ^4^Department of Radiology, Henan Provincial People's Hospital, Zhengzhou 450003, China; ^5^School of Cyber Science and Engineering, Zhengzhou University, Zhengzhou 450002, China; ^6^Hanwei IoT Institute, Zhengzhou University, Zhengzhou 450002, China

## Abstract

Accurate preoperative glioma grading is essential for clinical decision-making and prognostic evaluation. Multiparametric magnetic resonance imaging (mpMRI) serves as an important diagnostic tool for glioma patients due to its superior performance in describing noninvasively the contextual information in tumor tissues. Previous studies achieved promising glioma grading results with mpMRI data utilizing a convolutional neural network (CNN)-based method. However, these studies have not fully exploited and effectively fused the rich tumor contextual information provided in the magnetic resonance (MR) images acquired with different imaging parameters. In this paper, a novel graph convolutional network (GCN)-based mpMRI information fusion module (named MMIF-GCN) is proposed to comprehensively fuse the tumor grading relevant information in mpMRI. Specifically, a graph is constructed according to the characteristics of mpMRI data. The vertices are defined as the glioma grading features of different slices extracted by the CNN, and the edges reflect the distances between the slices in a 3D volume. The proposed method updates the information in each vertex considering the interaction between adjacent vertices. The final glioma grading is conducted by combining the fused information in all vertices. The proposed MMIF-GCN module can introduce an additional nonlinear representation learning step in the process of mpMRI information fusion while maintaining the positional relationship between adjacent slices. Experiments were conducted on two datasets, that is, a public dataset (named BraTS2020) and a private one (named GliomaHPPH2018). The results indicate that the proposed method can effectively fuse the grading information provided in mpMRI data for better glioma grading performance.

## 1. Introduction

Glioma is the most common primary brain tumor, which accounts for nearly 80% of all malignant brain tumors [1]. Generally, gliomas are categorized as low-grade gliomas (LGGs) and high-grade gliomas (HGGs). In a clinical setting, LGG patients have a good prognosis, while HGG patients often have a poor one. Therefore, treatment options for patients with different grades of gliomas are different. Currently, glioma grading is performed by pathological examinations of tumor tissues obtained by surgery. As a result, it is not possible to make personalized treatment plans before operation, and noninvasive glioma grading methods are urgently needed [2].

Multiparametric magnetic resonance imaging (mpMRI) is the most common imaging method for examining brain tumors and is very valuable for their diagnosis [3]. This imaging technology does not only reflect the information of human internal tissue noninvasively but also shows the tissue morphology, anatomical structure, contrast of different tissues, and other information of various imaging parameters in mpMRI of glioma. For instance, T1 can better reflect the anatomical structure, T1CE can distinguish the enhanced tumor and nonenhanced tumor according to the degree of blood flow, T2 provides the degree of peritumoral edema, and FLAIR can better reflect the anatomical information of the tumor by inhibiting the edema information [4]. Previous studies have shown that the information contained in mpMRI of patients with glioma has the potential for auxiliary grading diagnosis; still, it is difficult for clinicians to effectively quantify this information [5, 6]. Therefore, it is necessary to carry out a comprehensive analysis of glioma mpMRI, as well as fully explore and utilize the diagnostic information in the data.

In the field of computer vision, deep learning has achieved outstanding performance in medical image analysis tasks [7–9]. As a common deep learning network architecture, convolutional neural networks (CNNs) have demonstrated their powerful representation learning capabilities and have been frequently utilized in classification tasks [10, 11]. CNNs can extract numerous features from input images and achieve promising results. After comparing them with the features extracted utilizing engineered approaches, the CNN features can better reflect the characteristics of the input. Thus, they have better classification capabilities, higher applicability, and stronger generalization abilities. CNNs have also been adopted to automatically extract features from glioma MRI for noninvasive grading and have made progress in this field [12–19]. However, a limitation of the existing studies is that they fully rely on CNNs to extract the information without considering the specific characteristics of mpMRI data. For mpMRI, joint analysis of data acquired with different imaging sequences and sufficient information fusion should be conducted to achieve better classification performance. Besides, the relationship between image slices in a whole 3D volume should also be comprehensively explored.

A graph is a classical data representation format, which is composed of multiple vertices and edges. The vertices often represent samples, and the information in each vertex usually reflects a certain state of the sample. The edges generally contain the associated information of the connected samples. A graph convolutional network (GCN) transfers the structured convolution operation to unstructured graph data by constructing a graph. In this way, a more effective representation can be learned through information interaction between adjacent vertices [20–22]. The GCN has attracted more attention in various fields, including medical image analysis. Previous studies have tried to transform image data into a graph structure and adopted GCN to fuse information more effectively [23–28].

In this study, a novel GCN-based mpMRI information fusion module, which is named MMIF-GCN, is proposed for enhanced glioma grading performance. Specifically, we construct a graph according to the characteristics of mpMRI data of glioma patients. The vertices are defined as the extracted CNN features of different MR image slices, and the edges describe the positional relationships between slices in a 3D MR image. Our method introduces a learnable nonlinear transformation to the information interaction between adjacent vertices, which can capture more powerful contextual features and improve the glioma grading performance. The proposed method provides a new perspective for information fusion of mpMRI data. Furthermore, we conducted extensive experiments on two datasets (i.e., a public dataset named BraTS2020 and a private one named GliomaHPPH2018), while multiple baseline CNN architectures have been investigated. The proposed MMIF-GCN module can consistently provide better information fusion and achieve better glioma grading results.

The main contributions of this work are listed as follows:

1. We propose a novel GCN-based mpMRI information fusion module, MMIF-GCN. Particularly, GCN is used for the first time to fuse the contextual information of MR image slices and the complementary information of different MR imaging parameters.
2. Our method transforms mpMRI data into a graph according to the characteristics of the data. With the graph, the physical importance of information fusion is clarified. In the process of fusing the information of different MR image slices, a nonlinear representation learning step is introduced to improve the information quality, while maintaining the positional relationship between adjacent slices.
3. Extensive experiments have been conducted on two datasets, one public dataset and one private dataset. The proposed MMIF-GCN method can consistently improve the glioma grading performance of multiple CNN baseline models.

## 2. Related Work

In this section, we briefly review related works from two perspectives. In the first part, we introduce studies that focus on utilizing CNNs to extract features from MR images for glioma grading. In the second part, we discuss previous work on GCN-based image information fusion.

### 2.1. Application of CNN in Glioma Grading

Based on successful applications of CNN in natural image classification, many studies have tried to perform glioma grading with MRI data using CNN-based methods. We group these studies into three major categories according to two criteria: (1) whether mpMRI data are utilized, and (2) whether contextual information relationships between MR image slices are exploited.

The first category refers to studies that meet neither of the two criteria. These studies utilize MR data from only one sequence, and they did not consider the contextual information between image slices. For example, Decuyper et al. [12] used only T1CE-MRI data from the BraTS2017 dataset for model training, extracted features with VGG-11, and constructed a prediction model for glioma grading based on the random forest classification algorithm. Yang et al. [13] collected MRI data with 6 different imaging sequences, but they used only T1CE-MRI data to train the models (AlexNet and GoogLeNet) in their study for glioma grading. The focus of these studies was to verify the capability of CNNs in obtaining glioma grading-relevant information from MRI. However, they did not consider the specific characteristics of mpMRI data. Consequently, the grading performance is limited.

The second category includes studies that meet one of the criteria. These studies built glioma grading models by fusing context information of MR image slices or information of MR data acquired with different imaging parameters. Shahzadi et al. [14] proposed the long short-term memory (LSTM) module to fuse the slices' contextual information of glioma MRI. The FLAIR-MRI of 60 patients from the BraTS2015 dataset was used as training data, and the features extracted by AlexNet, ResNet, and VGGNet were inputted into the LSTM module to construct a grading model fused with slice context information. Ge et al. [15] proposed a CNN model using 3D convolution to extract context features between slices for glioma grading. The study used the T1CE-MRI sequence training model of 285 patients from the BraTS2017 dataset. Similarly, Mzoughi et al. [16] used a 3D CNN model to extract features and predict the grade of glioma from the T1CE-MRI of 285 patients from the BraTS2018 dataset. Zhuge et al. [17] collected a joint dataset of BraTS2018 and TCIA including MRI data with 4 parameters of 315 patients. The glioma grading model was constructed based on a Mask R-CNN. The slices of T1CE, T2, and FLAIR images were constructed into three-channel PNG data to achieve mpMRI fusion. Ge et al. [18] proposed a multistream CNN model to achieve information fusion of MRI images with different parameters. In the study, the features of 4 MR images from the BraTS2017 are extracted, and element-wise multiplication was used to realize the information fusion of images with various parameters. The fusion performance is better than that of the single MRI. In contrast to the first category of research work, these studies intentionally fuse context information of MR image slices or information of MR data acquired with different imaging parameters, but there is still room for improvement.

The third category contains studies that meet both criteria of fusing context information of MR image slices and information of MR data acquired with different imaging parameters. The study presented by Ye et al. [19] is based on a 3D CNN for extracting context information in MRI, and the information in different MRI sequences is fused by the designed module. The study was carried out for 274 patients from the BraTS2015 dataset. The experimental results show that the fusion of contextual information obtained from different MRI sequences can improve the prediction performance. Moreover, in comparison with simple information fusion, further improvement of the information fusion method can improve the performance of the proposed method. The method can only contain MRI of two parameters, so the amount of information that can be fused is limited.

Most of the aforementioned studies have tried to construct a glioma grading model based on the characteristics of mpMRI data; however, there are certain limitations in fully fusing the grading information of mpMRI. Our method realizes the fusion of mpMRI data characteristics through using graph convolution, which has advantages in fusing interactive information and improves the grading prediction performance of the CNN model.

### 2.2. Image Information Fusion with the Graph Convolutional Network

With the continuous development of methods for graph analytics, the application of these methods in the field of computer vision has also made major progress. Here, we introduce the research application of the GCN method in natural and medical images and analyze its role in practical applications.

For the analysis of natural images, some studies used GCN to realize information interaction and fusion in order to improve the performance of specific tasks. Li et al. [23] tried to use GCN as a new method to capture the long-distance context dependency between objects and other elements in a scene for the purpose of visual recognition research. In their study, the vertices of the graph are pixel clusters with similar characteristics. The edges are constructed according to the similarity of information between each vertex. Finally, the information interaction between the vertices of the graph is completed through the GCN, so as to capture the long-distance dependency of context and improve the recognition performance. Similarly, Xu et al. [24] transformed various objects in an image into graph data. Different objects in the graph constitute vertices and learned potential connections are edges from the characteristics of these objects. The information between co-occurrence and locations of objects in the process of image recognition is realized through the information interaction of the GCN, which helps to improve the performance of the model. Knyazev et al. [25] used a GCN to realize the classification task of natural image data. In this study, the image is transformed into superpixels of different scales as the vertices of the graph, and multiple edges are constructed according to the various relationships between the vertices. Then, a GCN is used to realize the interaction and fusion of information between vertices and, finally, improve the classification performance. It can be seen that these studies on natural image analysis have aimed at solving specific information fusion problems because of the use of GCN.

Additionally, there are some research studies using GCN fusion information for the analysis of medical images. Chen et al. [26] proposed a novel GCN framework, which can integrate the co-occurrence and interdependency of different pathological labels in chest X-ray images and improve the classification performance of the model. In this method, the vertex of the graph corresponds to the pathology, and the edge is the relationship between pathologies. Liu et al. [27] aimed at the problem that the complementary information of the mediolateral oblique and craniocaudal views of a mammogram are difficult to obtain using conventional methods, and they proposed a GCN-based method to achieve the interactive fusion of two modal information, which improves the performance and interpretability of the model. After obtaining the design of the research study, different regions in each view are vertices. The two types of views form two types of vertex sets. The edges between the two types of vertices are constructed through geometric and semantic relation learning. Tian et al. [28] used a GCN to achieve interactive segmentation of prostate MR images. The study used N vertices to form the prostate segmentation contour. The vertex information is the feature vector and position coordinates of the image, while the edge is the prostate segmentation contour formed by the connection of vertices. The interactive segmentation results are transmitted to all vertices through the graph convolutional vertex information fusion so that each vertex learns a new position information update and improves the accuracy of the overall segmentation. It can also be seen that the GCN method has research value in fusing medical image information.

So far, the aforementioned research studies have to design imaging data as graph data according to task requirements and, then, use GCN to realize the information interaction between vertices and adjacent vertices. In a similar way, our research study is aimed at characteristics of different images complementary information and organizational context information in glioma mpMRI data, so as to transform this information into graph data, clarify the physical meaning of the graph, and realize learnable information fusion.

## 3. Method

### 3.1. Overview

The architecture of our proposed module, MMIF-GCN, is shown in Figure 1. The architecture consists of feature extraction, graph construction, graph convolutional network, and classification. It is assumed that each glioma patient corresponds to MRI with 4 different imaging parameters, and the MRI of each parameter has *n* corresponding slices containing tumor information. *F*_*i*_^(*k*)^ represents the feature extracted by a CNN from the *i*^*th*^ MRI axial slice of the *k*^*th*^ parameter (*k* ∈ [1,4], *i* ∈ [1, *n*]). {*X*_*i*_}_*i*=1_^*n*^ represents the mpMRI feature vector learned by nonlinear mapping after feature concatenation of the *i*^*th*^ slice layer of k-parametric MRI. We combine the above information with the positional relationship of slices to present the graph *G*=(*𝒱*, *ℰ*), where *v*_*i*_ ∈ *𝒱* represents vertices, and the information of vertices *X*_*i*_ and (*v*_*i*_, *v*_*j*_) ∈ *ℰ* represents edges, reflecting the proximity relationship between different slices. We define the adjacency matrix as *A* ∈ *ℝ*^*n*×*n*^, the feature vectors matrix of the vertex as *X* ∈ *ℝ*^*n*×*D*^, where *D* represents the dimension of the feature after nonlinear mapping.

### 3.2. Feature Extraction

First, 2D slices containing tumor regions were obtained from MRI with different imaging parameters of glioma patients. Then, common CNN models are used to extract the tumor grading features in the slices. These models include AlexNet [29], VGGNet-16 [30], GoogLeNet-Inceptionv3 [31], ResNet-34 [32], EfficientNet-b3 [33]. When extracting features using AlexNet and VGGNet-16, the last pooling layer in the network is modified to global max pooling, and the pooled features are extracted as the final features used by the slice. When using ResNet-34 and GoogLeNet-Inceptionv3 to extract features, the features before the fully connected layer are used as the final features of the slice. When using EfficientNet-b3 to extract features, a global average pooling layer needs to be added after the last MBConvBlock, and the pooled features are used as the final features of the slice.

### 3.3. Graph Construction

The process for converting grading information of glioma extracted from mpMRI into a graph data structure is the key to realize information fusion through GCN. In this study, according to the characteristics of mpMRI data, the representation of the graph was designed. The details are described in the following.

Vertex represents a slice of a certain position of the tumor in the MRI of a glioma patient.

Vertex information: *X*_*i*_ represents the glioma grading information learned from the *i*^*th*^ MR slice. In our study, we used CNN to extract the glioma grading features from the same location slices of four parameters MRI which are represented by *F*_*i*_^(1)^, *F*_*i*_^(2)^, *F*_*i*_^(3)^, *F*_*i*_^(4)^. The integration of information in slices at the same position in mpMRI is achieved through the concatenation of feature matrices. In order to effectively fuse tumor grading information in images with different parameters, the dimensions of various extracted CNN features are unified. We have added a nonlinear encoder *f*. Through this learnable nonlinear representation, the effective fusion of different grading information is achieved and the dimensionality of the vertex information is unified. The following formula shows the fusion process of slice information at the same location in mpMRI:

(1) $$\begin{array}{c} X_{i}=f\left(\text{Concat}\left(F_{i}^{\left(1\right)},F_{i}^{\left(2\right)},F_{i}^{\left(3\right)},F_{i}^{\left(4\right)}\right)\right). \end{array}$$

Edge represents the edge between vertices, which reflects whether the positions of the slices are close in the MRI. We have taken into account the way that medical imaging specialists need to consider the information of several adjacent slices above and below when analyzing slices at a certain location. Then, we constructed edges between corresponding vertices of adjacent slices. We set each slice to be connected to the 3 adjacent slices above and below, and each vertex has a total of 6 edges. Based on the definition of the above edge, we construct the corresponding adjacency matrix. The definition of the adjacency matrix *A* ∈ *ℝ*^*n*×*n*^ is as follows:

(2) $$\begin{array}{c} A_{ij}=\left\{\begin{array}{cc} 1, & if\;\left|i-j\right|\leq 3,\\ \text{0}, & \text{otherwise}, \end{array}\right. \end{array}$$

where |*i* − *j*| represents the distance between the *i*^*th*^ and *j*^*th*^ slices.

### 3.4. Graph Convolutional Network

Graph convolution realizes the convolution operation in graph structures data through the information interaction between each vertex and adjacent vertices. The process consists of an aggregator and an updater. The aggregator can fuse the information contained in all vertices connected to the current vertex. The updater can fuse the current vertex information with the aggregated information of adjacent vertices and update the fused information into the vertices. Through the convolution operation on all vertices in the graph, the information fusion of each vertex and adjacent vertices is realized, and the fused vertex information is put into the corresponding vertices in the new graph with the same structure [20, 34]. To realize the dissemination and fusion of each vertex information through multiple GCN iterations, this learnable information fusion method can help the model to obtain a better feature representation.

The graph convolution method used in this research is shown in Figure 2. In this study, *G*_0_ represents the initial graph, and *X*_0_⟶*X*^″^ is the process of performing a graph convolution on a vertex. *X*_0_ represents the vertex information of the current graph convolution operation in the graph, and *X*_*i*_, *i* ∈ [1,6] represents the information in the 6 vertices connected to the vertex, where *X*_*i*_ ∈ *ℝ*^*D*^. The aggregator will first perform nonlinear mapping of *X*_*i*_ to obtain new information *X*_*i*_′, presented in formula (3), where *X*_*i*_′ ∈ *ℝ*^*D*^. Then, through the max pooling operation on *X*_*i*_′, *i* ∈ [1,6], the aggregate information *X*_*neigh*_^″^ is obtained, as shown in formula (4), where *X*_*neigh*_^″^ ∈ *ℝ*^*D*^. Subsequently, the updater concatenates *X*_0_ and *X*_*neigh*_^″^ to obtain *X*_*cat*_, where *X*_*cat*_ ∈ *ℝ*^2  *D*^, and then, uses nonlinear maps to obtain the final fused information *X*′′, as shown in formula (5), where *X*^″^ ∈ *ℝ*^*D*^. After all vertices in the graph perform graph convolution operation to fuse information, a new graph with the same structure and different information is obtained by using residual connection, as shown in formula (6).

(3) $$\begin{array}{c} X_{i}^{\prime }=\text{ReLU}\left(F\left(X_{i}\right)\right), \end{array}$$

(4) $$\begin{array}{c} X_{neigh}^{\prime \prime }=\text{MaxPooling}\left(X_{1},X_{2},X_{3},X_{4},X_{5},X_{6}\right), \end{array}$$

(5) $$\begin{array}{c} X^{\prime \prime }=\text{ReLU}\left(BN\left(F\left(\text{Concat}\left(X_{0},X_{\text{neigh}}^{\prime \prime }\right)\right)\right)\right), \end{array}$$

(6) $$\begin{array}{c} G_{n}=GCN\left(G_{n-1},w_{n-1}\right)+G_{n-1}, \end{array}$$

where *F*(·) represents a linear transformation using the fully connected network and then a nonlinear transformation through ReLU(·), MaxPooling(·) represents global max pooling, Concat(·) represents feature concatenation, and *BN*(·) represents batch normalization. *GCN*(·) represents a convolution operation for each vertex in the graph according to formulas (3)–(5). *w*_*n*−1_ represents the training parameters of the convolution operation in layer *n* − 1.

### 3.5. Global Average Pooling and Classification

After *n* iterations in order to update the initial graph, the graph after fusion information is finally obtained. The information of all vertices is merged into a one-dimensional feature vector through global average pooling, which is used as the input of the fully connected layer in the entire network. Finally, the network model achieves classification training using the softmax and cross-entropy loss functions.

## 4. Results and Discussion

### 4.1. Datasets

In this study, two datasets were used to evaluate the performance of the method, namely, the public dataset BraTS2020 and the private dataset GliomaHPPH2018 that were collected from the Henan Provincial People's hospital.  Figure 3 shows image examples of the two datasets. The specific details of the two datasets are described as follows.

BraTS2020: this dataset contains multiparametric glioma MRI data [35], and it is a public dataset that is widely used in glioma image analysis. This dataset was acquired with different clinical protocols and various scanners from multiple institutions. It contains 369 samples (293 HGG and 76 LGG). In our experiment, it was randomly shuffled into three subsets by the patient: 60% for training, 20% for validation, and 20% for testing.

GliomaHPPH2018: this dataset is derived from the PACS system of Henan Provincial People's Hospital (Henan, China) between 2012 and 2018. It contains 232 samples (157 HGG and 75 LGG). This study was approved by the local ethics committee. Given the retrospective nature of the study and the anonymity of patient data, the requirement for written informed consent was waived. Similarly, the GliomaHPPH2018 dataset was randomly shuffled into three subsets by the patient: 60% for training, 20% for validation, and 20% for testing.

Lastly, all data met the following criteria: (1) preoperative images were obtained, including T1CE, T1, T2, and FLAIR sequences; (2) the histopathological examination and grading of gliomas were in accordance with WHO criteria.

### 4.2. Experimental Setting

First, the slices obtained from different CNN models have different feature dimensions. To unify the input information dimensionality of the MMIF-GCN module and reduce the number of model parameters, we set the features of mpMRI slices to 200 through the encoder, that is, *X*_*i*_ ∈ *ℝ*^200^. The number of iterations for each graph is 4 (i.e., *G*_0_⟶*G*_4_).

The proposed model is implemented using PyTorch [36] and the DGL [37] framework and runs on GeForce RTX 2080Ti GPU with 12 GB memory. In our experiment, the batch size is set to 16, and the initial learning rate is set to 5 × 10^−6^. When the network performance is not improved within 10 epochs, the learning rate is reduced by half. In addition, we adjust the size of the original image to 224 × 224. During training, we use the Adam optimizer to train 200 epochs through the cross-entropy loss function.

### 4.3. Effectiveness of Information Fusion Using MMIF-GCN

This study uses accuracy and the area under the receiver operating characteristic curve (AUC) as evaluation indices to compare the classification performance of different models. The experiment was carried out based on the MRI data with 4 different parameters from the BraTS2020 and GliomaHPPH2018 datasets. The effectiveness of the proposed method in the fusion of MRI slice context information and MRI complementary information of different imaging parameters is verified.

To demonstrate the effectiveness of graph convolution methods in helping common CNN models to fuse contextual information, this study compares the tumor grading performance of common CNN models for each parameter MRI and the performance of GCN as a contextual information fusion module. The experimental results are shown in Table 1. We found that all CNN models can use GCN to fuse MRI slice context information to improve the classification performance of the model. At the same time, we compared the performance of the context information fusion method based on graph convolution and 3D convolution, as shown in Table 2. To eliminate the influence of network structure on model performance, we uniformly choose CNN that is based on the ResNet framework as the training model to compare performances. The experimental results show that the contextual information fusion method based on graph convolution has more potential to improve the classification performance of the model for different parameters MRI.

In addition, Table 1 shows that our proposed MMIF-GCN can simultaneously fuse slice context information and MRI complementary information for different imaging parameters, as well as improve the performance of common CNN models in glioma grading tasks. Similarly, Table 3 shows the performance of our MMIF-GCN method and the other two models that can simultaneously fuse different parameters MRI complementary information and slice context information. The experimental procedures of these two methods are shown in Figure 4. N(1) represents a glioma grading model that uses 3D convolution to fuse context information and concatenates feature information to fuse complementary MRI information with different parameters. N(2) represents a model built by fusing each parameter MRI with graph convolution to fuse context information and, then, concatenate the final features to fuse multiparametric MRI information. The results indicate that our proposed MMIF-GCN module can fuse better the grading information in mpMRI of glioma patients, as well as predict better the tumor grade of patients. We speculate that this is due to the well-designed MMIF-GCN fusion method, which adds learnable nonlinear representation to each 2D mpMRI information fusion process, while considering the context information. Therefore, the effect is better than directly concatenating and analyzing the information of MRI with different parameters. This result is similar to the conclusion of the study carried out by Ye et al. [19].

### 4.4. Ablation Studies

In this section, we evaluate the impact of parameters on grading results based on two aspects, that is, the vertex feature dimensionality of GCN and the number of graph iterations that are described as follows:

Vertex feature dimensions of GCN: the model needs to select the smallest feature dimensionality to accurately express the information of the original feature. After fixing other parameters, we set a series of different vertex feature dimensions for the MMIF-GCN (i.e., {50, 100, 200, 300}) to evaluate the performance separately. As shown in Figure 5, when the vertex feature dimensionality is set to 200, our proposed MMIF-GCN achieves the best performance on both datasets and each network framework.

The number of iterations of GCN in the graph is an important issue in the GCN-related research. Thus, it is necessary to ensure effective information interaction but also prevent the smoothness of multiple iterations. In our experiment, we set the number of iterations of GCN in the graph to *m*, where *m* ∈ [2,5]. As shown in Figure 6, after 4-layer GCN iterations and fusion of information, our proposed MMIF-GCN module achieved the best performance on both datasets and each network framework.

## 5. Conclusions

In this study, we propose a novel GCN-based mpMRI information fusion module, named MMIF-GCN. With this module, an effective fusion of contextual information extracted from 2D mpMRI slices can be accomplished, and enhanced glioma grading performance can be achieved. Extensive experiments on two datasets utilizing multiple baseline CNN models have been conducted, and the effectiveness of the proposed method for the information fusion of mpMRI data has been properly validated.

There are several limitations to our study. In terms of clinical problems, only glioma grading was studied. In further studies, we will try to apply the MMIF-GCN method to the aided diagnosis analysis in 3D multiparameter medical images of other diseases to further verify the effectiveness of the proposed method. Methodologically, this study was limited to the fusion of features extracted from 2D CNN models. In the future, we will try to add the 2D slice features extracted by the radiomics method for feature fusion.

## Figures and Tables

**Figure 1:** Overview of the proposed framework.

**Figure 2:** The process of graph convolution operation.

**Figure 3:** Image examples of 4-sequence MRI from BraTS2020 and GliomaHPPH2018 datasets.

**Figure 4:** Methodology for realizing mpMRI context and multiparameter information fusion simultaneously. (a) N(1). (b) N(2).

**Figure 5:** Classification accuracy of the validation set under different CNN models and vertex feature dimensionality of GCN. (a) BraTS2020 dataset. (b) GliomaHPPH2018 dataset.

**Figure 6:** Classification accuracy of the validation set under different CNN models and GCN iterations. (a) BraTS2020 dataset. (b) GliomaHPPH2018 dataset.

**Table 1:** Demonstration of the graph convolution module can fuse contextual information in MRI with different imaging parameters to improve the performance of the CNN models.

Dataset	Method	GoogLeNet-Inceptionv3		EfficientNet-b3		ResNet-34		AlexNet		VGGNet-16	
		AUC	ACC	AUC	ACC	AUC	ACC	AUC	ACC	AUC	ACC
BraTS2020	T1CE	0.911	0.893	0.921	0.893	0.932	0.907	0.910	0.880	0.915	0.867
	**G-TICE**	**0.931**	**0.907**	**0.936**	**0.920**	**0.946**	**0.920**	**0.943**	**0.907**	**0.947**	**0.893**
	T1	0.851	0.813	0.884	0.867	0.896	0.840	0.804	0.800	0.854	0.827
	**G-T1**	**0.860**	**0.853**	**0.896**	**0.880**	**0.906**	**0.853**	**0.816**	**0.827**	**0.863**	**0.853**
	T2	0.893	0.867	0.892	0.853	0.849	0.840	0.867	0.853	0.876	0.840
	**G-T2**	**0.904**	**0.893**	**0.904**	**0.893**	**0.873**	**0.880**	**0.886**	**0.880**	**0.903**	**0.880**
	FLAIR	0.897	0.827	0.885	0.853	0.894	0.853	0.802	0.827	0.889	0.840
	**G-FLAIR**	**0.911**	**0.867**	**0.905**	**0.867**	**0.908**	**0.867**	**0.834**	**0.840**	**0.915**	**0.867**
	**MMIF-GCN**	**0.963**	**0.920**	**0.974**	**0.933**	**0.986**	**0.947**	**0.954**	**0.933**	**0.974**	**0.920**

GliomaHPPH2018	T1CE	0.810	0.787	0.952	0.851	0.842	0.787	0.802	0.809	0.867	0.787
	**G-TICE**	**0.904**	**0.851**	**0.965**	**0.894**	**0.900**	**0.830**	**0.846**	**0.830**	**0.929**	**0.872**
	T1	0.898	0.872	0.923	0.872	0.921	0.894	0.729	0.766	0.933	0.872
	**G-T1**	**0.913**	**0.894**	**0.942**	**0.915**	**0.962**	**0.915**	**0.821**	**0.830**	**0.942**	**0.936**
	T2	0.692	0.766	0.798	0.745	0.729	0.745	0.629	0.660	0.856	0.766
	**G-T2**	**0.769**	**0.787**	**0.856**	**0.851**	**0.813**	**0.787**	**0.731**	**0.809**	**0.863**	**0.830**
	FLAIR	0.873	0.809	0.967	0.872	0.931	0.872	0.838	0.766	0.879	0.851
	**G-FLAIR**	**0.890**	**0.830**	**0.973**	**0.915**	**0.942**	**0.894**	**0.846**	**0.809**	**0.896**	**0.872**
	**MMIF-GCN**	**0.960**	**0.936**	**1.000**	**0.979**	**0.996**	**0.979**	**0.881**	**0.851**	**0.979**	**0.957**

*Note. G* means to fuse context information with GCN. The results of our study are shown in bold.

**Table 2:** Demonstration of the context information fusion method based on graph convolution and 3D convolution.

Dataset	Method	T1CE		T1		T2		FLAIR	
		AUC	ACC	AUC	ACC	AUC	ACC	AUC	ACC
BraTS2020	2D-ResNet	0.932	0.907	0.896	0.840	0.849	0.840	0.894	0.853
	3D-ResNet	0.939	0.920	0.905	0.853	0.860	0.880	0.853	0.867
	**G-2D-ResNet**	**0.946**	**0.920**	**0.906**	**0.853**	**0.873**	**0.880**	**0.908**	**0.867**

GliomaHPPH2018	2D-ResNet	0.842	0.787	0.921	0.894	0.729	0.745	0.931	0.872
	3D-ResNet	0.844	0.809	0.960	0.894	0.750	0.766	0.923	0.872
	**G-2D-ResNet**	**0.900**	**0.830**	**0.962**	**0.915**	**0.813**	**0.787**	**0.942**	**0.894**

**Table 3:** The performance of three methods of fusing mpMRI context and multiparameter information in two different datasets is compared.

Dataset	Method	Base-ResNet	
		AUC	ACC
BraTS2020	N(1)	0.949	0.920
	N(2)	0.970	0.920
	**MMIF-GCN**	**0.986**	**0.947**

GliomaHPPH2018	N(1)	0.965	0.894
	N(2)	0.969	0.936
	**MMIF-GCN**	**0.996**	**0.979**

The results of our study are shown in bold.

## Data Availability

The datasets used in this paper are the public dataset BraTS2020 and Henan Provincial People's Hospital dataset GliomaHPPH2018; BraTS2020 can be obtained through the following URL: https://www.kaggle.com/awsaf49/brats20-dataset-training-validation.

## References

[1] Filippini G. (2012). Epidemiology of primary central nervous system tumors. *Handbook of Clinical Neurology*.

[2] Sengupta A., Ramaniharan A. K., Gupta R. K., Agarwal S., Singh A. (2019). Glioma grading using a machine‐learning framework based on optimized features obtained from T 1 perfusion MRI and volumes of tumor components. *Journal of Magnetic Resonance Imaging*.

[3] Bauer S., Wiest R., Nolte L.-P., Reyes M. (2013). A survey of MRI-based medical image analysis for brain tumor studies. *Physics in Medicine and Biology*.

[4] Tan Y., Zhang S.-t., Wei J.-w. (2019). A radiomics nomogram may improve the prediction of IDH genotype for astrocytoma before surgery. *European Radiology*.

[5] Zhao G., Man P., Bai J. (2021). AI-powered radiomics algorithm based on slice pooling for the glioma grading. *IEEE Transactions on Industrial Informatics*.

[6] Tian Q., Yan L.-F., Zhang X. (2018). Radiomics strategy for glioma grading using texture features from multiparametric MRI. *Journal of Magnetic Resonance Imaging*.

[7] Zhou S. K., Greenspan H., Davatzikos C. (2021). A review of deep learning in medical imaging: imaging traits, technology trends, case studies with progress highlights, and future promises. *Proceedings of the IEEE*.

[8] Liu X., Yuan Q., Gao Y. (2022). Weakly supervised segmentation of COVID-19 infection with scribble annotation on CT images. *Pattern Recognition*.

[9] He J., Zhu Q., Zhang K., Yu P., Tang J. (2021). An evolvable adversarial network with gradient penalty for COVID-19 infection segmentation. *Applied Soft Computing*.

[10] Yang Y., Hu Y., Zhang X., Wang S. (2021). Two-stage selective ensemble of CNN via deep tree training for medical image classification. *IEEE Transactions on Cybernetics*.

[11] Sun Y., Xue B., Zhang M., Yen G. G., Lv J. (2020). Automatically designing CNN architectures using the genetic algorithm for image classification. *IEEE Transactions on Cybernetics*.

[12] Decuyper M., Bonte S., Van Holen R. Binary glioma grading: radiomics versus pre-trained CNN features.

[13] Yang Y., Yan L.-F., Zhang X. (2018). Glioma grading on conventional MR images: a deep learning study with transfer learning. *Frontiers in Neuroscience*.

[14] Shahzadi I., Tang T. B., Meriadeau F., Quyyum A. CNN-LSTM: cascaded framework for brain Tumour classification.

[15] Ge C., Qu Q., Gu I. Y.-H., Jakola A. S. 3D multi-scale convolutional networks for glioma grading using MR images.

[16] Mzoughi H., Njeh I., Wali A. (2020). Deep multi-scale 3D convolutional neural network (CNN) for MRI gliomas brain tumor classification. *Journal of Digital Imaging*.

[17] Zhuge Y., Ning H., Mathen P. (2020). Automated glioma grading on conventional MRI images using deep convolutional neural networks. *Medical Physics*.

[18] Ge C., Gu I. Y.-H., Jakola A. S., Yang J. Deep learning and multi-sensor fusion for glioma classification using multistream 2D convolutional networks.

[19] Ye F., Pu J., Wang J., Li Y., Zha H. Glioma grading based on 3D multimodal convolutional neural network and privileged learning.

[20] Kipf T. N., Welling M. Semi-supervised classification with graph convolutional networks.

[21] Zhou J., Cui G., Hu S. (2020). Graph neural networks: a review of methods and applications. *AI Open*.

[22] Hamilton W. L., Ying R., Leskovec J. Inductive representation learning on large graphs.

[23] Li Y., Gupta A. Beyond grids: learning graph representations for visual recognition.

[24] Xu H., Jiang C., Liang X., Li Z. Spatial-aware graph relation network for large-scale object detection.

[25] Knyazev B., Lin X., Amer M. R., Taylor G. W. Image classification with hierarchical multigraph networks.

[26] Chen B., Li J., Lu G., Yu H., Zhang D. (2020). Label co-occurrence learning with graph convolutional networks for multi-label chest x-ray image classification. *IEEE journal of biomedical and health informatics*.

[27] Liu Y., Zhang F., Zhang Q., Wang S., Wang Y., Yizhou Y. Cross-view correspondence reasoning based on bipartite graph convolutional network for mammogram mass detection.

[28] Tian Z., Li X., Zheng Y. (2020). Graph-convolutional-network-based interactive prostate segmentation in MR images. *Medical Physics*.

[29] Krizhevsky A., Sutskever I., Hinton G. E. (2017). ImageNet classification with deep convolutional neural networks. *Communications of the ACM*.

[30] Simonyan K., Zisserman A. Very deep convolutional networks for large-scale image recognition.

[31] Szegedy C., Liu W., Jia Y. Going deeper with convolutions.

[32] He K., Zhang X., Ren S., Sun J. Deep residual learning for image recognition.

[33] Tan M., Le Q. Efficientnet: rethinking model scaling for convolutional neural networks.

[34] Wu Z., Pan S., Chen F., Long G., Zhang C., Yu P. S. (2020). A comprehensive survey on graph neural networks. *IEEE Transactions on Neural Networks and Learning Systems*.

[35] Menze B. H., Jakab A., Bauer S. (2014). The multimodal brain tumor image segmentation benchmark (BRATS). *IEEE Transactions on Medical Imaging*.

[36] Paszke A., Gross S., Massa F. Pytorch: an imperative style, high-performance deep learning library.

[37] Wang M., Yu L., Zheng D. Deep graph library: towards efficient and scalable deep learning on graphs.

